# Comparative Analysis of Deepfake Image Detection Method Using Convolutional Neural Network

**DOI:** 10.1155/2021/3111676

**Published:** 2021-12-16

**Authors:** Hasin Shahed Shad, Md. Mashfiq Rizvee, Nishat Tasnim Roza, S. M. Ahsanul Hoq, Mohammad Monirujjaman Khan, Arjun Singh, Atef Zaguia, Sami Bourouis

**Affiliations:** ^1^Department of Electrical and Computer Engineering, North South University, Dhaka 1229, Bangladesh; ^2^School of Computing and IT, Manipal University Jaipur, Jaipur, Rajasthan, India; ^3^Department of Computer Science, College of Computers and Information Technology, Taif University, Taif 21944, Saudi Arabia; ^4^Department of Information Technology, College of Computers and Information Technology, Taif University, P.O. Box 11099, Taif 21944, Saudi Arabia

## Abstract

Generation Z is a data-driven generation. Everyone has the entirety of humanity's knowledge in their hands. The technological possibilities are endless. However, we use and misuse this blessing to face swap using deepfake. Deepfake is an emerging subdomain of artificial intelligence technology in which one person's face is overlaid over another person's face, which is very prominent across social media. Machine learning is the main element of deepfakes, and it has allowed deepfake images and videos to be generated considerably faster and at a lower cost. Despite the negative connotations associated with the phrase “deepfakes,” the technology is being more widely employed commercially and individually. Although it is relatively new, the latest technological advances make it more and more challenging to detect deepfakes and synthesized images from real ones. An increasing sense of unease has developed around the emergence of deepfake technologies. Our main objective is to detect deepfake images from real ones accurately. In this research, we implemented several methods to detect deepfake images and make a comparative analysis. Our model was trained by datasets from Kaggle, which had 70,000 images from the Flickr dataset and 70,000 images produced by styleGAN. For this comparative study of the use of convolutional neural networks (CNN) to identify genuine and deepfake pictures, we trained eight different CNN models. Three of these models were trained using the DenseNet architecture (DenseNet121, DenseNet169, and DenseNet201); two were trained using the VGGNet architecture (VGG16, VGG19); one was with the ResNet50 architecture, one with the VGGFace, and one with a bespoke CNN architecture. We have also implemented a custom model that incorporates methods like dropout and padding that aid in determining whether or not the other models reflect their objectives. The results were categorized by five evaluation metrics: accuracy, precision, recall, *F*1-score, and area under the ROC (receiver operating characteristic) curve. Amongst all the models, VGGFace performed the best, with 99% accuracy. Besides, we obtained 97% from the ResNet50, 96% from the DenseNet201, 95% from the DenseNet169, 94% from the VGG19, 92% from the VGG16, 97% from the DenseNet121 model, and 90% from the custom model.

## 1. Introduction

The face is the most distinctive feature of human beings. With the tremendous growth of face synthesis technology, the security risk posed by face manipulation is becoming increasingly significant. Individuals' faces may often be swapped with someone else's faces that appear authentic because of the myriads of algorithms based on deep learning technology. Deepfake is an emerging subdomain of artificial intelligence technology in which one person's face is overlaid over another person's face. More specifically, multiple methods based on generative adversarial networks (GANs) produce high-resolution deepfake images [1]. Unfortunately, due to the widespread usage of cellphones and the development of numerous social networking sites, deepfake content is spreading faster than ever before in the twenty-first century, which has turned into a global danger [2]. Initially, deepfake images were discernible with the human eye due to the pixel collapse phenomena that tend to create artificial visual inconsistencies in the skin tone or facial shape of pictures. Not only images or videos, but also audio can be turned into deepfakes. Deepfakes have grown to be barely distinguishable from natural pictures as technology has progressed over the years [3]. Consequently, people all across the world are experiencing inescapable complications.

Because of deepfake technology, people may choose their fashion more quickly, which benefits the fashion and e-commerce industries. Furthermore, this technology aids the entertainment business by providing artificial voices for artists who cannot dub on time. Additionally, filmmakers can now recreate many classic sequences or utilize special effects in their films because of deepfake technology. Deepfake technology can potentially let Alzheimer's patients communicate with a younger version of themselves, which might help them retain their memories. GANs are also being investigated for their application in detecting anomalies in X-ray images [4]. The deepfake approaches often require a massive quantity of image, video, or audio data to generate natural photos so that the witnesses are persuaded to believe them. Besides all the prominence, there are some significant drawbacks as well. Public figures, for instance, celebrities, athletes, and politicians, are the worst sufferers of deepfakes as they have a substantial number of videos and pictures available online. Though deep fake technologies are occasionally used to ridicule others, they are primarily employed to create adulterous content. The faces of many celebrities and other well-known individuals have been grafted onto the bodies of pornographic models, and these images are widely available on the Internet [2]. Deepfake technology may create satirical, pornographic, or political content about familiar people by utilizing their pictures and voices without their consent. Due to the ease of various applications, anyone can fabricate any artificial content imperceptible to the actual content [2]. Many young people are becoming victims of cyberbullying. In the worst-case scenario, countless sufferers commit suicide.

A deep fake video of the former American president Barack Obama is being circulated on the Internet these days where he is uttering things that he has never expressed. Furthermore, deepfakes have already been used to alter Joe Biden's footage showing his tongue out during the US 2020 election. Besides, Taylor Swift, Gal Gadot, Emma Watson, Meghan Markle, and many other celebrities have been victims of deepfake technology [5]. In the United States and Asian societies, many women are also victimized by deep fake technologies. The harmful use of deep fakes can significantly impact our culture and increase misleading information, especially on social media [6]. However, because of the negative impacts on different individuals and organizations, deepfakes have been a significant threat to our current generation. Therefore, to eradicate defamation, scams, deception, and insecurities from society, researchers have been relentlessly trying to detect deepfakes. The identification of deepfakes would reduce the number of crimes that are currently occurring around the world. Therefore, researchers have paid attention to the mechanism for validating the integrity of deepfakes [2]. In reaction to this trend, some multinational companies have started to take initiatives. For instance, Google has made a fake video database accessible for academicians to build new algorithms to detect deepfake, while Facebook and Microsoft have organized the Deepfake Detection Challenge [7].

There are several methods to detect GAN-generated deepfake images, including the traditional machine learning classifiers (Support Vector Machine Algorithm, or naive algorithms), deep neural networks, convolutional neural networks (CNN), recurrent neural networks (RNN), long short-term memory (LSTM), and many more. The main contribution of the work is to identify the deepfake images and distinguish them from the normal images using CNN architecture. In this research, eight different architectures using convolutional neural networks have been employed to detect deepfake images, including DenseNet169, DenseNet121, DenseNet201, VGG16, VGG19, VGGFace, and ResNet50. A custom model has also been introduced to do comparative analysis.

The dataset for this work was obtained from Kaggle. At its commencement, the dataset was gathered. Hence, the features have been extracted, and various CNN architectures have been implemented to obtain the best result. Finally, each model was evaluated using four different metrics: accuracy, precision, recall, and *F*1-score. Lastly, the area under the ROC curve was also considered another metric for assessing the performance of the models.

## 2. Related Works

While deepfake is a relatively new technology, there has been research done on the topic. Nguyen et al. and his colleagues performed a study [2] that examined the use of deep learning to create and detect deepfakes. The number of deepfake articles has grown significantly in recent years, according to data gathered by https://app.dimensions.ai towards the end of 2020. Although the number of deepfake articles acquired is likely to be lower than the exact amount, the research trend on this issue is rising. The capacity of deep learning to represent complex and high-dimensional data is well-known. Deep autoencoders, a type of deep network having such an ability, have been widely used for dimensionality reduction and picture compression [8–10].

The FakeApp, developed by a Reddit user utilizing an autoencoder-decoder pairing structure, was the first effort at deepfake generation [11, 12]. The autoencoder collects latent characteristics from facial pictures, and the decoder reconstructs the images in that way. Two encoder-decoder pairs are required to switch faces between source and target pictures; the encoder's parameters are shared between two network pairs, and each pair is used to train on an image collection. The encoder networks of these two pairs are identical [2]. This method using the encoder-decoder architecture is used in several recent types of research, including DeepFaketf (TensorFlow-based deepfakes) [13], DFaker [14], and DeepFaketf (TensorFlow-based deepfakes) [15]. An enhanced version of deepfakes based on the generative adversarial network (GAN) [10], for example, face swap-GAN, was suggested in [16] by adding the adversarial loss and perceptual loss to the encoder-decoder architecture, as implemented in VGGFace [17].

Furthermore, the FaceNet implementation [18] introduces a multitask convolutional neural network (CNN) to improve face identification and alignment reliability. The CycleGAN [19] is used to construct generative networks. Deepfakes are posing a growing threat to privacy, security, and democracy [20]. As soon as the risks of deepfakes were identified, strategies for monitoring them were developed. In recent approaches, deep learning automatically extracts significant and discriminative characteristics to detect deepfakes [21, 22]. Korshunov and Marcel [23, 24] used the open-source code Faceswap-GAN [19] to create a unique deepfake dataset containing 620 videos based on the GAN model to address this issue. Low and high-quality deepfake films were made using videos from the publicly accessible VidTIMIT database [25], efficiently imitating facial expressions, lip movements, and eye blinking. According to test findings, the popular facial recognition algorithms based on VGG and Facenet [18, 26] are unable to identify deepfakes efficiently. Because deep learning algorithms like CNN and GAN can improve legibility, facial expression, and lighting in photos, swapped face images have become harder for forensics models [27]. To create fake photos with a size of 128 × 128, the large-scale GAN training models for high-quality natural image synthesis (BIGGAN) [28], self-attention GAN [27], and spectral normalization GAN [29] are employed. On the contrary, Agarwal and Varshney [30] framed the GAN-based deepfake detection problem as a hypothesis testing problem, using a statistical framework based on the information-theoretic study of authenticity [31].

When used to detect deepfake movies from this newly created dataset, other methods such as lip-syncing approaches [32–34] and picture quality measures with support vector machine (SVM) [35] generate very high error rates. To get the detection results, the extracted features are put into an SVM classifier. In their paper [36], Zhang et al. utilized the bag of words approach to extract a collection of compact features, which they then put into classifiers like SVM [37], random forest (RF) [38], and multilayer perceptron (MLP) [39] to distinguish swapped face images from real ones. To identify deepfake photos, Hsu et al. [40] proposed a two-phase deep learning technique. The feature extractor in the first phase is based on the common fake feature network (CFFN), and it leverages the Siamese network design described in [41]. To leverage temporal differences across frames, a recurrent convolutional model (RCN) was suggested based on the combination of the convolutional network DenseNet [42] and the gated recurrent unit cells [43]. The proposed technique is evaluated on the FaceForensics++ dataset [44], which contains 1,000 videos, and shows promise. Guera and Delp [45] have pointed out that deepfake videos include intraframe discrepancies and temporal anomalies between frames. They then proposed a temporal-aware pipeline technique for detecting deepfake films that employs CNN and long short-term memory (LSTM).

Deepfakes have considerably lower blink rates than regular videos. To distinguish between actual and fake videos, Li et al. [46] deconstructed them into frames, extracting face regions and eye areas based on six eye landmarks. These cropped eye landmark sequences are distributed into long-term recurrent convolutional networks (LRCN) [47] for dynamic state prediction after a few preprocessing stages, such as aligning faces, extracting and scaling the bounding boxes of eye landmark points to produce new sequences of frames. To identify fake photos and videos, Nguyen et al. [48] recommended using capsule networks. The capsule network was created to overcome the constraints of CNNs when employed for inverse graphics tasks [49], which attempt to discover physical processes that form pictures of the environment. The ability of a capsule network based on a dynamic routing algorithm [50] to express hierarchical pose connections between object components has recently been observed. They include the Idiap Research Institute replay-attack dataset [51], Afchar et al. deepfake's face-swapping dataset [52], the facial reenactment FaceForensics dataset [44], developed by the Face2Face technique [53], and Rahmouni et al. entirely computer-generated picture dataset [54].

Researchers in [55] advocated using photo response nonuniformity (PRNU) analysis to distinguish genuine deepfakes from fakes. PRNU is sometimes regarded as the digital camera's fingerprint left in the photos [56]. Because the swapped face is intended to affect the local PRNU pattern in the facial area, the analysis is frequently utilized in picture forensics [57–60] and is proposed for use in [57]. The goal of digital media forensics is to create tools that allow for the automated analysis of a photo or video's integrity. In this research, both feature-based [61, 62] and CNN-based [63, 64] integrity analysis techniques have been investigated. Raghavendra et al., in their paper [65], suggested using two pretrained deep CNNs to identify altered faces, while Zhou [66] recommended using a two-stream network to detect two distinct face-swapping operations. A recent dataset by Rössler [67], which contains half a million altered pictures created with feature-based face editing, will be of particular interest to practitioners.

Then the paper is organized as follows: Section 2 discussed the influential works on detecting deepfake images. Then, the techniques employed in our research are described in Section 3. In Section 4, the results are presented, and comparative analysis is carried out. Finally, Section 5 draws the paper to a conclusion.

The main objective of this paper is to efficiently distinguish deepfake images from normal images. There have been a lot of studies done on the delicate issue of “'deepfake.” Many researchers used a CNN-based strategy to identify deepfake images, while others used feature-based techniques. To detect the deepfake images, few of them used machine learning classifiers. But the novelty of this work is that it is able to detect deepfake images from normal images with 99% accuracy using the VGGFace model. We implemented more CNN architectures in our study than many other researchers, which has distinguished our work. A comprehensive analysis has been demonstrated in our work, and the outcome outperformed previous work.

## 3. Methodology

Figure 1 presents the fundamental diagram of several deep learning architectures. At the outset, the dataset was collected, and the features were extracted. Hence, eight deep learning architectures have been employed that were evaluated against five different evaluation metrics, including accuracy, precision, *F*1-score, recall, and the area under the ROC curve.

In Figure 1, the input is first obtained from a dataset collected from Kaggle and then sent through the convolution layer. This layer extracts numerous characteristics from the input photos. Convolution is a mathematical process that is conducted between the input picture and a filter of specified size (P × P). The dot product between the filter and the input image portion is calculated by sliding the filter across the image (P × P). The resulting feature map provides information about the image's corners and edges. This feature map is later used by additional layers to learn more about the input picture.

Afterward, it passes through the pooling layer. The main goal of this layer is to minimize the size of the convolved feature map. This is accomplished by reducing the connections between layers and operating independently on each feature map. Diverse methods of pooling provide distinct results. Max-pooling selects the biggest element from the feature map. Average pooling determines the average of the items included within a set image section size.

It then passes through the fully connected layer. The fully connected (FC) layer connects two layers of neurons. It has the weights, biases, and neurons. Input from the previous levels is flattened and sent to the FC layer. Further FC layers are utilized to conduct mathematical functional operations on the flattened vector. This stage initiates the categorization process.

### 3.1. Data

The dataset was acquired from Kaggle, which included 70,000 real faces from the Flickr dataset collected by Nvidia Corporation. Besides, there were 70,000 fake faces out of the one million fake faces that were produced by styleGAN. Later, both of the datasets were combined, and the images were resized to 256 pixels. Lastly, the dataset was divided into three parts, including the train, validation, and test set. There were 100000 images in the training set, with 50000 images being real and the rest being fake. In the validation set, there were 20,000 images, of which 10,000 were real, and the rest were fake. Finally, the other 20000 images were equally divided into real and fake in the test set.

Deepfake image detection is a complicated method that takes several aspects into account. The fundamental procedures for imaging classification will include the identification of an appropriate classification scheme, training sample collection, image preprocessing, extraction of features, selection, and accuracy evaluation of appropriate grade methods. The core deepfake framework includes the use of generative adversarial networks [2], generative models that learn how to distribute their data without any supervision. The Kaggle dataset utilized in this research, “140k Real and Fake Faces,” consists of 70000 fake faces prepared by styleGAN [68]. We have trained 8 CNN models for this comparative research of the usage of CNN networks to classify real and deepfake images. Three of the models that were trained are of the DenseNet architecture (DenseNet121, DenseNet169, and DenseNet201), two are of the VGGNet architecture (VGG16, VGG19), one is using the ResNet50 architecture, one is using the VGGFace, and one is with a custom CNN architecture. Each model is discussed at length in the following sections.

### 3.2. Proposed Network

Convolutional neural networks are constructed by using numerous smaller units of neurons that take place in a layered fashion. The neurons are then connected with each other, and the edges that connect them have weight. The weights of the training model are updated every epoch using techniques like backpropagation. A convolutional neural network consists of two portions. The first one is the feature extraction portion, and the second one is the classification portion. We used pretrained networks such as DenseNet, which exists in the Keras API.  Figure 2 shows the architecture of DenseNet. We have used different versions of the DenseNet (e.g., DenseNet201, DenseNet169, and DenseNet121) pretrained model to improvise the prediction results. It is a convolutional network that is connected layer in a feedforward fashion. Each layer gets new inputs from all preceding levels and passes them on to all following layers to maintain the feedforward nature [42].

### 3.3. Dense Blocks

A convolutional layer is a fundamental building block of a neural network. A fixed size is used to extract the complex features of the given data. The DenseNet convolution network is divided into multiple dense blocks. For example, in the DenseNet169 architecture, there are 169 layers in 4 dense blocks. Apart from that, there are 3 transition layers, 1 classification layer, and 1 convolutional layer. The dense blocks consist of 6, 12, 32, and 32 convolutional layers. The initial convolution of the architecture is 112 × 112, followed by a max-pooling of 56 × 56. The model input is a blob that takes each image input of 1 × 3 × 224 × 224 in BGR order.

### 3.4. DenseNet121

Dense convolutional network (DenseNet) is a widespread expansion of the Residual CNN (ResNet) architecture. DenseNet differentiates by providing an immediate connection between each layer and all subsequent network layers instead of its ResNet and other convolution neural networks [42]. We wanted to keep in mind that the DenseNet121 model in Keras is accurate, with a bit of tweaking using a dense layer as the final layer. The model consisted of four dense blocks of closely related layers, such as Batch Standardization (BN) and 3 × 3 turnaround. Moreover, the pattern also featured a transition layer between every dense block with an average pooling layer of 2 × 2 and a concentration of 1 × 1. We inserted the customized dense layer with the sigmoid activation after the last dense block.

### 3.5. DenseNet201

Due to the ability to feature reuse by successive layers, the DenseNet201 uses a condensed network, enabling easy-to-train and parametrically efficient models. This increases the variety of the succeeding layer input and enhances performance [42].

### 3.6. DenseNet169

DenseNet169 contains 169 layers of depth, a minimal number of parameters compared to other models, and has better handling of the vanishing gradient problem.

Besides, ResNet50 is implemented in this work to observe the evaluation metrics.  Figure 3 shows the architecture of ResNet50. ResNet, short for Residual Network, is a neural network developed to tackle a complicated issue by stacking more layers in deep neural networks, resulting in increased accuracy and performance. Adding more layers is based on the idea that these layers will learn increasingly complicated characteristics.

### 3.7. ResNet50

ResNet50 is a familiar ResNet variation of 48 convolution layers, 1 max-pool layer, and 1 average pool layer. There are 3.8 × 109 floating-point operations in it.

### 3.8. VGG16

The most distinctive feature of VGG16 is that, rather than having a massive number of hyperparameters, they concentrated on having 3 × 3 filter convolution layers with a stride of 1 and always utilized the same padding and max-pool layer as the 2 × 2 filter stride 2.  Figure 4 shows the architecture of VGG16. Throughout the design, the convolution and max-pool layers are arranged in the same way. It features two fully connected layers at the end, followed by a softmax for output. The 16 in VGG16 alludes to the fact that it contains 16 layers with different weights [71].

### 3.9. VGG19

VGG19 is a convolutional neural network model with several convolutional layers and nonlinear activation layers that outperforms a single convolutional layer.  Figure 5 shows the architecture of VGG19. The layer structure allows for improved image feature extraction, downsampling using max-pooling, and modification of the rectified linear unit (ReLU) as the activation function, which selects the greatest value in the image region as the pooled value of the area. The downsampling layer is primarily used to increase the network's antidistortion capabilities of the picture while preserving the sample's primary characteristics and lowering the number of parameters.

### 3.10. VGGFace

VGGFace is an image recognition model that produces the most advanced outputs from Oxford's Visual Geometry Group researchers' standard datasets for face recognition [74]. This technique allows us to build a large data set for training while utilizing only a modest amount of annotation power.  Figure 6 shows the architecture of VGGFace. We used the VGGFace architecture proposed by Tai Do Nhu and Kim [73] to build the model. This model included five blocks of the layer, with convolutional and max-pooling layers in each block. Two 3 × 3 convolution layers followed by a pooling layer were each in the first and second block. Three 3 × 3 convolution layers, each composed of the third, fourth, and fifth blocks, are followed by a max-pooling layer. The ReLU activation function was employed in all convolutional layers. Since VGGFace uses pretrained weights, we have had to adapt to our needs. After the five-layer blocks that gave us the facial characteristics, we fine-tuned them by adding dense layers. Finally, the output layer with sigmoid activation was also included as a dense layer.

Lastly, a custom model has been introduced to this work to see the overall variation, as shown in Figure 7.

### 3.11. Custom CNN

This model helps to determine whether the other models are as good as they promise. Figure 7 shows the architecture of the custom model. This model also includes techniques such as dropout and padding, which are not included in the other models. We can study whether such strategies improve CNN's performance. We have employed six convolutional layers for the custom design, each paired with batch normalization and max-pooling layers. For all convolutional layers, the activation function was the rectified linear unit (ReLU). We also used dropout to decrease the fit for every convolutional layer. We employed padding to allow the kernel to have more room to check the image, thus increasing the precision of the image as well as dropouts. As this was a binary classification task, we added a dense layer at the end with sigmoid activation on top of the convolutional base.

## 4. Results and Analysis

This comparative study showed that convolutional neural networks are highly effective in the detection and classification of GAN-generated images. The performance of the models has been assessed with five different metrics: accuracy, precision, recall, *F*1-score, and area under the ROC curve.

### 4.1. Confusion Matrix

A confusion matrix of size *n* × *n* (*n* number of rows and columns) associated with a classifier shows the predicted and actual classification, where *n* is the number of different classes. For *n* × *n* matrices, True Positive (TP), True Negative (TN), False Negative (FN), and False Positive (FP) are calculated using the following equations [75]:

(1) $$\begin{array}{c} {\text{TP}}_{i}=a_{ii},\\ {\text{FP}}_{i}=\sum_{j=1,j\neq i}^{n}a_{ji},\\ {\text{FN}}_{i}=\sum_{j=1,j\neq i}^{n}a_{ij},\\ {\text{TN}}_{i}=\sum_{j=1,j\neq i}^{n}\sum_{k=1,k\neq i}^{n}a_{jk}. \end{array}$$

Here, predictions can be correct or wrong. The confusion matrix for DenseNet121 is illustrated in Figure 8. From the confusion matrix, 9480 fake images and 9926 real images were correctly classified by the network. However, 520 fake images were classified as real and 74 real images were classified as fake images.

The confusion matrix for DenseNet201 has been shown in Figure 9. Unlike the aforementioned DenseNet121 model, DenseNet201 has performed better in terms of identifying fake images, which is 9503. Even though there is no significant difference, the model has not been able to identify real images as it has misclassified 138 real images as fake and 497 fake images as real.

The confusion matrix for DenseNet169 has been shown in Figure 10. The confusion matrix for DenseNet169 has been shown in Figure 10. It has identified 9758 images as fakes out of the 10000 fake images. On the other hand, 9751 real images were identified as real correctly, whereas it misclassified 249 real images as fake and 242 fake images as real.

Figure 11 represents the confusion matrix for ResNet50. The model misclassified a total of 494 images. 9824 fake images and 9682 real images were correctly classified.

Figure 12 depicts the confusion matrix for VGG16. The VGG16 model identified 9619 fake images correctly. On the other hand, it failed to classify 1693 real images as real. 8307 real images were correctly identified, and 381 fake images were misclassified.

The confusion matrix for VGG19 is shown in Figure 13. 9426 fake images were successfully classified as fake images, and 9435 real images were classified as real images. On the contrary, the model classified 574 fake images as real and 565 real images as fake.

Figure 14 illustrates the confusion matrix for VGGFace. The model correctly classified 9916 real images and 9835 fake images. On the contrary, only fake images and 165 real images were misclassified.

Finally, the confusion matrix for the custom model is shown in Figure 15. 168 fake images were misclassified. Also, 1522 real images were classified as fake. 9832 fake images and 8478 real images were classified correctly.

### 4.2. Accuracy

The number of times correct estimates are made is referred to as accuracy. Accuracy is calculated using the following equation:

(2) $$\begin{array}{c} \text{accuracy}=\frac{\text{number of correct predictions}}{\text{total number of predictions made}}. \end{array}$$

It only works best if each class has an equal number of samples.

### 4.3. Precision

Precision, also known as positive predictive value, refers to how well the model predicts positive values out of all the positive values predicted by the model. The term “precision” refers to the following:

(3) $$\begin{array}{c} \text{precision}=\frac{\text{True Positive}}{\text{True Positive}+\text{False Positive}}. \end{array}$$

### 4.4. Recall

Recall can be used to measure how well the model detects true positives. A high recall is an indicator that the model has done well at identifying true positives. On the contrary, if the recall value is low, the model encounters many false negatives. The term “recall” refers to the following:

(4) $$\begin{array}{c} \text{recall}=\frac{\text{True Positive}}{\text{True Positive}+\text{False Negative}}. \end{array}$$

### 4.5. *F*1-Score

It is the harmonic mean of precision and recall. The *F*1-score provides a better estimate than the accuracy metric of the wrongly categorized cases.

(5) $$\begin{array}{c} F1\;-\text{score}=2\frac{\text{Precision}}{\text{Precision}+\text{Recall}}. \end{array}$$

The *F*1-score is required to balance precision and recall. We saw before that True Negatives contribute a great deal to accuracy. The *F*1-score may be a better measure if we need to balance precision and recall and there is an uneven class distribution (a large number of Actual Negatives) [76].

### 4.6. Receiver Operating Characteristic Curve (ROC) and Area under the ROC Curve (AUC)

For classification tasks, the AUC-ROC curve is used to assess the algorithm's performance. ROC is the probability curve, and AUC indicates the degree or level of separability. It shows how well the model can differentiate between classes. In general, the AUC indicates how well the model predicts 0 and 1 classes correctly. For example, the greater the AUC is, the more accurate the model discriminates between patients with and without illness. Let us first define some terms.

The receiver operating characteristic (ROC) curve illustrates the relationship between True Positive Rate and False Positive Rate at various categorization levels. Reduce the categorization threshold, and more items are classified as positive, increasing both False Positives and True Positives [77].

An AUC of around 1 indicates that a model is excellent, suggesting a high degree of separability. An inadequate model has an AUC value close to zero, meaning that it has the lowest measure of separability. Indeed, it implies that the outcome is reciprocated. It is mistaking 0 s for 1 s and 1 s for 0 s. And an AUC of 0.5 indicates that the model has no capability for class differentiation at all.

### 4.7. Model Accuracy and Loss

The training accuracy, validation accuracy, training loss, and validation loss graphs for all the models are illustrated in Figures 16(a) and 16(b).

#### 4.7.1. DenseNet121

Training accuracy, validation accuracy, training loss, and validation loss graphs for DenseNet121 are shown.

In Figure 16, the given graph on the left side shows us training accuracy and validation accuracy over the course of 10 epochs for the model DenseNet121. We can observe that training accuracy steadily improved and reached nearly 100%, whereas validation accuracy rose and subsequently fluctuated and reached a point where the gap between training and validation accuracy was minimal. Similarly, training loss dropped progressively over time, whereas validation loss decreased first and then fluctuated. The overfitting problem was observed after the training crossed the 10 epoch mark. On the contrary, training loss dropped progressively over time, whereas validation loss decreased first till the 2nd epoch and then fluctuated during the 3rd, 6th, and 9th epochs with an increasing loss score of more than 0.1 at least.

#### 4.7.2. DenseNet169

Training accuracy, validation accuracy, training loss, and validation loss graphs for DenseNet169 are illustrated underneath in Figures 17(a) and 17(b).

In Figure 17, the graph on the left side illustrates the training and validation accuracy of the model DenseNet169 over the course of 10 epochs. We can observe that training accuracy grew steadily, but validation accuracy increased but fluctuated after the eighth period, before increasing again. Training accuracy almost touched the 100% mark, whereas validation accuracy touched the 95% mark. The model started at a training and testing accuracy of 70% and crossed the 90% mark. Training loss dropped progressively, but validation loss reduced gradually but varied after the eighth epoch, reaching above 0.6 before decreasing again to just above 0.1 on the 10th epoch.

#### 4.7.3. DenseNet201

Training accuracy, validation accuracy, training loss, and validation loss graphs for DenseNet201 are given in Figures 18(a) and 18(b).

As displayed in Figure 18, the graph on the left side illustrates the training and validation accuracy of the model DenseNet201 over the course of 10 epochs. The training accuracy seems to improve as the epochs increase. However, the validation accuracy has some fluctuations over the time period. At the third epoch, the validation accuracy dropped below 50%. However, by the 10th epoch, the results were touching the 96% score. The training loss was quite constant over epochs, while the validation loss rose, then fell, and remained rather steady, touching 0, across the remaining epochs.

#### 4.7.4. VGG16

Training accuracy, validation accuracy, training loss, and validation loss graphs for VGG16 are shown in Figures 19(a) and 19(b).

As shown in Figure 19, the graph on the left side depicts the training and validation accuracy of the model VGG16 over the course of 10 epochs. The training accuracy and validation accuracy seem to have a steady rise as the epochs increase. The graph on the right side depicts the training and validation loss of the model over the period of 10 epochs, reaching below 0.2.

#### 4.7.5. VGG19

Training accuracy, validation accuracy, training loss, and validation loss graphs for VGG19 are illustrated in Figures 20(a) and 20(b).

In Figure 20, the graph on the left side illustrates the training and validation accuracy of the model VGG19 over the course of 10 epochs. Both the training accuracy and the validation accuracy seem to have a steady rise as the epochs increase, achieving more than 90%. The graph on the right side depicts the training and validation loss of the model over the period of 10 epochs and reaching the 0.1 loss mark.

#### 4.7.6. VGGFace

The graphs for VGGFace's training accuracy, validation accuracy, training loss, and validation loss are shown in Figures 21(a) and 21(b).

Figure 21 displays the plot for training and validation accuracy and training and validation loss for our best-resulting model compared to other models in our experiment. The validation accuracy of the model trains the data with more than 95% accuracy on every epoch, eventually reaching an impressive 99% validation accuracy. Additionally, the training and validation loss decrease to close to the 0 mark.

#### 4.7.7. ResNet50

Training accuracy, validation accuracy, training loss, and validation loss graphs are given in Figures 22(a) and 22(b).

As shown in Figure 22, the pretrained architecture of ResNet50 shows that it has more training and validation accuracy than most other pretrained models in 2 or 3 epochs. The training accuracy of ResNet50 reaches over 95%. However, the validation accuracy reached 97%. While training loss dropped steadily, validation loss decreased smoothly until the third epoch and then varied.

#### 4.7.8. Custom CNN

Training accuracy, validation accuracy, training loss, and validation loss graphs for custom CNN are shown in Figures 23(a) and 23(b).

Finally, in Figure 23, the accuracy and loss of our proposed custom model are plotted. Even though the training accuracy of the model has a steady rise, the validation accuracy has some fluctuations over the course of the 10 epochs. While training loss dropped steadily, validation loss decreased smoothly until the second epoch and then varied. The model does not show promising results as far as validation accuracy is concerned. However, it still reaches the 90% mark.

### 4.8. Model Evaluation

Table 1 illustrates the findings received from all the CNN architectures.

Finally, Figure 24 shows the comparison amongst all the models that have been implemented in this work. Amongst all the pretrained convolutional architectures, VGGFace achieved an impressive 99% accuracy on our training set. On the other hand, the least performed architecture, VGG16, achieved 92% accuracy. DenseNet121 and ResNet50 achieved the same accuracy of 97%, which is the second best performing model. DenseNet201 and DenseNet169 achieved an accuracy of 96% and 95%, respectively. The highest precision score of 99% was achieved by four models. The models are VGGFace, DenseNet169, DenseNet121, and ResNet50. However, only VGGFace could achieve the best result in recall, which is 98%. The second best models, achieving close to the score of VGGFace, were the DenseNet201 and the VGG19 models, which achieved 97% recall. The *F*1-score of the VGGFace architecture was the highest, reaching an impressive 99%. The lowest *F*1-score was achieved by DenseNet121, as the *F*1-score was only 82%. The second best model, according to the *F*1-score, was ResNet50, as it achieved a 97% *F*1-score. The highest AUC score was 99.8%, achieved by the VGGFace architecture, and the lowest was achieved by the DenseNet121 architecture. The custom model proposed by the authors achieved 90% accuracy on the dataset. The custom architecture achieved 84% precision and the highest score in terms of recall. The *F*1-score fell down to 91% even though the recall score was 99%. A decent AUC score of 98.9% was achieved as well.

A bar graph was generated using Table 1. The graphical representation of the table shows us the exact scores as a whole. Evidently, VGGFace performed best in every category, achieving the best score amongst all the pretrained networks. However, the custom model achieved a 99% recall score, which is the highest score amongst all the recall scores of other pretrained architectures. ResNet50 was the second best architecture, obtaining a 97% *F*1-score. Overall, the least performing architecture was DenseNet121, which achieved only 82% *F*1-score as it scored only 70% on recall.

### 4.9. Model Comparison

Table 2 shows a comparison graph of several works that have been examined by deepfake. Table 2 contrasts this paper with several other studies completed by other researchers using the same models that we utilized in our research. Studies [78, 79] used VGG19 and VGG16, respectively, and the corresponding accuracies were 80.22% and 81.6%, respectively. The authors of the study [42] used several DenseNet models to conduct their research, and the accuracies for DenseNet169, DenseNet201, and DenseNet121 were 93.15%, 93.66%, and 92.29%, respectively. The authors of the research also used ResNet50, where the accuracy was 81.6%.

### 4.10. Model Test

The precision of our study was further clarified by some more experiments. The experiment was done by providing fake and real images of each of the models. Almost all of the pictures were correctly identified or classified as “real” or “fake” as shown in Figure 25. From the validation directory, as many as ten pictures were randomly selected from each of the original and deepfake images.

## 5. Conclusion and Future Work

Deepfake is an emerging technology that is being used to deceive a large number of people. Though not all deepfake contents are malicious, they need to be detected since some of the deepfake contents are indeed threatening to the world. The primary purpose of this study was to find a reliable and accurate way to detect deepfake images. Many other researchers have been working relentlessly to detect deepfake content using a variety of methodologies. The significance of this work, however, is that it achieves excellent results using CNN architecture. This study uses eight CNN architectures to detect deepfake images from a large dataset. The results have been reliable and accurate. VGGFace performed the best in several metrics, including accuracy, precision, *F*1-score, and area under the ROC curve. However, in terms of recall, the custom model implemented in the study performed slightly better than the VGGFace. The results of the custom models, DenseNet169, DenseNet201, VGG19, VGG16, ResNet50, and DenseNet121, were impressive as well. Finally, collected deepfake images have been analyzed to detect whether they are deepfakes or not, where the result is satisfactory.

This breakthrough work will have a tremendous impact on our society. Using this technology, deepfake victims can quickly determine whether the pictures are real or fake. People will remain vigilant since they will have the capability to identify the deepfake image through our work. In the future, we may apply the CNN algorithms to a video deepfake dataset for the convenience of many sufferers.

Many other experiments and tests have been left for future work. We aim to collect real data from our local community and classify deepfake images from normal images using a convolutional neural network. We may apply more efficient models to identify the deepfake images to reduce crime in our society and, moreover, in our world. We believe our contribution will eventually aid in the reduction of unwanted suicide cases and blackmail in our society.

## Figures and Tables

**Figure 1:** Workflow diagram.

**Figure 2:** Architecture of DenseNet [69].

**Figure 3:** Architecture of ResNet50 [70].

**Figure 4:** Architecture of VGG16 [72].

**Figure 5:** Architecture of VGG19 [73].

**Figure 6:** Architecture of VGGFace [74].

**Figure 7:** Architecture of the custom model.

**Figure 8:** The confusion matrix for DenseNet121.

**Figure 9:** The confusion matrix for DenseNet201.

**Figure 10:** The confusion matrix for DenseNet201.

**Figure 11:** The confusion matrix for ResNet50.

**Figure 12:** The confusion matrix for VGG16.

**Figure 13:** The confusion matrix for VGG19.

**Figure 14:** The confusion matrix for VGG face.

**Figure 15:** The confusion matrix for custom CNN.

**Figure 16:** DenseNet121 training and validation accuracy and loss.

**Figure 17:** DenseNet169 training and validation accuracy and loss.

**Figure 18:** DenseNet201 training and validation accuracy and loss.

**Figure 19:** VGG16 training and validation accuracy and loss.

**Figure 20:** VGG19 training and validation accuracy and loss.

**Figure 21:** VGGFace training and validation accuracy and loss.

**Figure 22:** ResNet50 training and validation accuracy and loss.

**Figure 23:** Custom CNN training and validation accuracy and loss.

**Figure 24:** Comparison graph amongst the model.

**Figure 25:** Screenshot of classification of the “real” and “fake” images.

**Table 1:** Obtained results after implementing the models.

CNN architecture's name	Accuracy	Precision	Recall	*F*1-score	AUC
VGG19	0.94	0.91	0.97	0.94	0.987
VGG16	0.92	0.93	0.92	0.92	0.977
VGGFace	0.99	0.99	0.98	0.99	0.998
DenseNet169	0.95	0.99	0.92	0.95	0.996
DenseNet201	0.96	0.96	0.97	0.96	0.994
DenseNet121	0.97	0.99	0.70	0.82	0.971
ResNet50	0.97	0.99	0.95	0.97	0.997
Custom model	0.90	0.84	0.99	0.91	0.989

**Table 2:** Comparison chart.

Reference	Model name	Accuracy (%)	Accuracy in this paper (%)
In study [78]	VGG19	80.22	94
In study [79]	VGG16	81.6	92
In study [42]	DenseNet169	93.15	95
In study [42]	DenseNet201	93.66	96
In study [42]	DenseNet121	92.29	97
In study [79]	ResNet50	81.6	97

## Data Availability

The data used to support the findings of this study are freely available at https://www.kaggle.com/xhlulu/140k-real-and-fake-faces.

## References

[1] Goodfellow I. J., Abadie J. P., Mirza M. (2014). Generative adversarial nets, “NIPS” 14. *Proceedings of the 27^th^ International Conference on Neural Information Processing Systems*.

[2] Nguyen T., Nguyen Q., Nguyen C. M., Nguyen D., Nguyen D., Nahavandi S. (2019). Deep learning for deepfakes creation and detection: a survey. https://arxiv.org/abs/1909.11573.

[3] Jung T., Kim S., Kim K. (2020). DeepVision: deepfakes detection using human eye blinking pattern. *IEEE Access*.

[4] Westerlund M. (2019). The emergence of deepfake technology: a review. *Technology Innovation Management Review*.

[5] Maras M.-H., Alexandrou A. (2019). Determining authenticity of video evidence in the age of artificial intelligence and in the wake of Deepfake videos. *International Journal of Evidence and Proof*.

[6] Almars A. M. (2021). Deepfakes detection techniques using deep learning: a survey. *Journal of Computer and Communications*.

[7] Guarnera L., Giudice O., Battiato S. DeepFake detection by analyzing convolutional traces.

[8] Punnappurath A., Brown M. S. (2020). Learning raw image reconstruction-aware deep image compressors. *IEEE Transactions on Pattern Analysis and Machine Intelligence*.

[9] Cheng Z., Sun H., Takeuchi M., Katto J. (2020). Energy compaction-based image compression using convolutional AutoEncoder. *IEEE Transactions on Multimedia*.

[10] Chorowski J., Weiss R. J., Bengio S., van den Oord A. (2019). Unsupervised speech representation learning using WaveNet autoencoders. *IEEE/ACM Transactions on Audio, Speech, and Language Processing*.

[11] Faceswap Deepfakes software for all. https://github.com/deepfakes/faceswap.

[12] https://www.malavida.com/en/soft/fakeapp/.

[13] DeepFaketf Deepfake based on tensorflow. https://github.com/StromWine/DeepFake%20tf.

[14] https://github.com/dfaker/df.

[15] https://github.com/iperov/DeepFaceLab.

[16] https://github.com/shaoanlu/faceswap-GAN.

[17] Keras-VGGFace VGGFace implementation with Keras frame-work. https://github.com/rcmalli/keras-vggface.

[18] https://github.com/davidsandberg/facenet.

[19] https://github.com/junyanz/pytorch-CycleGAN-and-pix2pix.

[20] Danielle Citron K., Chesney R. (2019). Deep fakes: a looming challenge for privacy, democracy, and national security, 107 California law review. https://scholarship.law.bu.edu/faculty_scholarship/640.

[21] De Lima O., Franklin S., Basu S., Karwoski B., George A. (2020). Deepfake detection using spatiotemporal convolutional networks. https://arxiv.org/abs/2006.14749.

[22] Amerini I., Caldelli R. Exploiting pre- diction error inconsistencies through LSTM-based classifiers to detect deepfake videos.

[23] Korshunov P., Marcel S. Vulnerability assessment and detection of deepfake videos.

[24] http://conradsanderson.id.au/vidtimit/.

[25] Parkhi O. M., Vedaldi A., Zisserman A. Deep face recognition.

[26] Schroff F., Kalenichenko D., Philbin J. Facenet: a unified embedding for face recognition and clustering.

[27] Zhang H., Goodfellow I., Metaxas D., Odena A. (2018). Self-attention generative adversarial networks. https://arxiv.org/abs/1805.08318.

[28] Brock A., Donahue J., Simonyan K. (2018). Large scale GAN training for high fidelity natural image synthesis. https://arxiv.org/abs/1809.11096.

[29] Miyato T., Kataoka T., Koyama M., Yoshida Y. (2018). Spectral normalization for generative adversarial networks. https://arxiv.org/abs/1802.05957.

[30] Agarwal S., Varshney L. R. (2019). Limits of deep- fake detection: a robust estimation viewpoint. https://arxiv.org/abs/1905.03493.

[31] Maurer U. M. (2000). Authentication theory and hypothesis testing. *IEEE Transactions on Information Theory*.

[32] Chung J. S., Senior A., Vinyals O., Zisserman A. Lip reading sentences in the wild.

[33] Suwajanakorn S., Seitz S. M., Kemelmacher-Shlizerman I. (2017). Synthesizing Obama. *ACM Transactions on Graphics*.

[34] Korshunov P., Marcel S. Speaker inconsistency detection in tampered video.

[35] Galbally J., Marcel S. Face anti-spoofing based on general image quality assessment.

[36] Zhang Y., Zheng L., Thing V. L. Automated face swapping and its detection.

[37] Wang X., Thome N., Cord M. (2017). Gaze latent support vector machine for image classification improved by weakly supervised region selection. *Pattern Recognition*.

[38] Bai S. (2017). Growing random forest on deep convolutional neural networks for scene categorization. *Expert Systems with Applications*.

[39] Zheng L., Duffner S., Idrissi K., Garcia C., Baskurt A. (2016). Siamese multi-layer perceptrons for dimensionality reduction and face identification. *Multimedia Tools and Applications*.

[40] Hsu C.-C., Zhuang Y.-X., Lee C.-Y. (2020). Deep fake image detection based on pairwise learning. *Applied Sciences*.

[41] Chopra S. Learning a similarity metric discriminatively, with application to face verification.

[42] Huang G., Liu Z., Van Der Maaten L., Weinberger K. Q. Densely connected convolutional networks.

[43] Cho K., van Merrienboer B., Gulcehre C. Learning phrase representations using RNN encoder–decoder for statistical machine translation.

[44] Rossler A., Cozzolino D., Verdoliva L., Riess C., Thies J., Nießner M. Faceforensics++: learning to detect manipulated facial images.

[45] Guera D., Delp E. J. Deepfake video detection using recurrent neural networks.

[46] Li Y., Chang M. C., Lyu S. Ictu oculi: exposing AI created fake videos by detecting eye blinking.

[47] Donahue J., Anne Hendricks L., Guadarrama S. Long- term recurrent convolutional networks for visual recognition and description.

[48] Nguyen H. H., Yamagishi J., Echizen I. Capsule-forensics: using capsule networks to detect forged images and videos.

[49] Hinton G. E., Krizhevsky A., Wang S. D. Transforming auto-encoders.

[50] Sabour S., Frosst N., Hinton G. E. (2017). Dynamic routing between capsules. *Advances in Neural Information Processing Systems*.

[51] Chingovska I., Anjos A., Marcel S. On the effectiveness of local binary patterns in face anti-spoofing.

[52] Afchar D., Nozick V., Yamagishi J., Echizen I. MesoNet: a compact facial video forgery detection network.

[53] Thies J., Zollhofer M., Stamminger M., Theobalt C., Nießner M. Face2Face: real-time face capture and reenactment of RGB videos.

[54] Rahmouni N., Nozick V., Yamagishi J., Echizen I. Distinguishing computer graphics from natural images using convolution neural networks.

[55] Koopman M., Rodriguez A. M., Geradts Z. Detection of deepfake video manipulation.

[56] Rosenfeld K., Sencar H. T. (2009). A study of the robustness of PRNU-based camera identification. *Media Forensics and Security International Society for Optics and Photonics*.

[57] Li C. T., Li Y. (2012). Color-decoupled photo response non-uniformity for digital image forensics. *IEEE Transactions on Circuits and Systems for Video Technology*.

[58] Lin X., Li C. T. (2017). Large-scale image clustering based on camera fingerprints. *IEEE Transactions on InformaTion Forensics and Security*.

[59] Scherhag U., Debiasi L., Rathgeb C., Busch C., Uhl A. (2019). Detection of face morphing attacks based on PRNU analysis. *IEEE Transactions on Biometrics, Behavior, and Identity Science*.

[60] Phan Q.-T., Boato G., De Natale F. G. B. (2019). Accurate and scalable image clustering based on sparse representation of camera fingerprint. *IEEE Transactions on Information Forensics and Security*.

[61] Sencar H. T., Memon N. (2013). *Digital Image Forensics*.

[62] Farid H. (2016). *Photo Forensics*.

[63] Güera D., Wang Y., Bondi L., Bestagini P., Tubaro S., Delp E. J. A counter forensic method for CNN-based camera model identification.

[64] Güera D., Yarlagadda S. K., Bestagini P., Zhu F., Tubaro S., Delp E. J. Reliability map estimation for cnn-based camera model attribution.

[65] Raghavendra R., Raja K. B., Venkatesh S., Busch C. Transferable deep-cnn features for detecting digital and print-scanned morphed face images.

[66] Zhou P. Two-stream neural networks for tampered face detection.

[67] Rössler A. (2018). Faceforensics: a large-scale video dataset for forgery detection in human faces. https://arxiv.org/abs/1803.09179.

[68] https://www.kaggle.com/xhlulu/140k-real-and-fake-faces.

[69] https://arxiv.org/abs/1608.06993.

[70] https://www.kaggle.com/keras/resnet50.

[71] https://towardsdatascience.com/step-by-step-vgg16-implementation-in-keras-for-beginners-a833c686ae6c.

[72] https://www.kaggle.com/shivamb/cnn-architectures-vgg-resnet-inception-tl.

[73] Tai Do Nhu I. N., Kim S. H. (2018). Forensics face detection from GANs using convolutional neural network. https://arxiv.org/abs/1902.11153v2.

[74] https://sefiks.com/2018/08/06/deep-face-recognition-with-keras/.

[75] Junayed M. S. AcneNet-a deep CNN based classification approach for acne classes.

[76] Accuracy P. Recall or *F*1. https://towardsdatascience.com/accuracy-precision-recall-or-f1-331fb37c5cb9.

[77] Classification ROC curve and AUC. https://developers.google.com/machine-learning/crash-course/classification/roc-and-auc.

[78] Gong D., Jaya Kumar Y., Goh O. S., Ye Zi, Chi W. (2021). DeepfakeNet, an efficient deepfake detection method. *International Journal of Advanced Computer Science and Applications (IJACSA)*.

[79] Tolosana R., Vera-Rodriguez R., Fierrez J., Morales A., Ortega-Garcia J. (2020). Deepfakes and beyond: a Survey of face manipulation and fake detection. *Information Fusion*.

